RETRACTED

# Income Gap Equalization Based on PSO Algorithm in Edge Computing Environment

**DOI:** 10.1155/2022/8316982

**Published:** 2022-08-10

**Authors:** Xiaomeng Zhao, Lin Liu

**Affiliations:** School of Economics and Management, Shihezi University, Xinjiang Shihezi 832000, China

## Abstract

In order to explore the current income gap, a method based on the PSO algorithm in the edge computing environment is proposed. PSO calculates and simulates bird flock foraging activities, the Frank Heppner biological group model, and the three rules in bird activities. After studying the activities of these natural creatures, abstract problems are quantified and similar models established. The Gini coefficient is calculated by using grouped data, and the grouping basis is also innovative. The quantile grouping method is adopted, which can effectively solve the difference between the concentration index and the Gini coefficient, and the Gini coefficients of each year can be added up to finally get the Gini coefficient of the stock income. Experimental results show that the Gini coefficient of traffic income in 2017 and 2018 had dropped significantly, but the variation of the Gini coefficient of stock income (Delta CG) was still greater than 0. Obviously, the adjustment speed of the Gini coefficient of stock income was lagging behind, as was the Gini coefficient of traffic income. We found that after 1986, the facilitation effect was greater than the dilution effect, and the facilitation effect continued to push up the stock income gap, which indicated more income flow to the high-income group, with the income flow gap showing an upward trend and the upward trend becoming more and more obvious. It has been proved that the PSO algorithm can effectively identify the income gap in the edge computing environment, and the corresponding policy suggestions are given.

## 1. Introduction

With the development of the economy, the development of various industries has an increasing demand for electric energy, which also makes the related technologies of the electric power industry develop rapidly. A stable and reliable power system is the key basis for the transmission and use of electrical energy, so the development of a stable power system is crucial to economic and social development [1]. The components of the power system involve many aspects, but the main ones can be divided into four parts, namely, users, power generation, power transmission, and power distribution. There are three main working modes: long-distance power transmission, centralized power generation, and large grid interconnection. While traditional power systems have some benefits, in many ways, they also have some drawbacks. First of all, in terms of the stability of power system operations, the traditional power system involves a relatively large area, so a small problem during the operation of the system may lead to power supply failure of the entire power system, resulting in large-scale power supply problems. In terms of system investment cost, a power system needs to pay a huge economic cost from the establishment of the system to the use and postmaintenance, and for such a huge project, postmaintenance is also very difficult; on the other hand, in some remote areas of the country with harsh natural environment, in order to operate the power system similarly, the need to invest more economic costs makes the final benefits even more unsatisfactory [2].

RETRACTED

As shown in Figure 1, edge computing is the core technology in current IoT applications. Edge computing completes real-time data processing on the edge side through the service capabilities of edge devices and edge servers. At the same time, edge servers provide services for different users and edge devices through the virtualized environment of container technology. These provide computing service offloading capability and, with the help of container technology, do not need to consider the environment configuration of the program and the security issues of resource isolation, which increases the flexibility of IoT applications. However, for the edge computing environment, its hardware resources (CPU, memory, disk, network, etc.) are usually limited [3]. How to efficiently manage and schedule container applications in the edge computing environment is the current big problem facing the application services. At present, the mainstream cloud service vendors usually use Kubernetes container cluster management tools to manage and schedule container applications. Since the design goal of the Kubernetes container cluster management tool is to manage large-scale container applications in the cloud computing environment, a simple and stable static scheduling algorithm is used in the scheduling algorithm; however, when this algorithm is used for the resource-constrained environment of edge computing, there are significant limitations. The particle swarm optimization (PSO) algorithm, proposed by two American doctors in 2002, is an evolutionary calculation method based on swarm intelligence, which can be used to solve a large number of nonlinear, nondifferentiable, nonconvex, high-dimensional complex optimization problems [4]. The optimization technique of the PSO algorithm can generate high-quality solutions in a short computing time and has more stable convergence characteristics than other random search methods. But its disadvantage is that its attempts can easily fall into the local minimum point, and the search accuracy is not high.

RETRACTED

## 2. Literature Review

The European Telecommunications Standards Institute (ETSI) proposed the concept of mobile edge computing (MEC), which integrates edge computing into the mobile network architecture. In 2016, Wi-Fi was connected on the basis of the original network, and the Chinese interpretation of MEC was changed to “multiaccess edge computing.” Computing offloading is an important research direction in MEC, which mainly includes offloading decision-making and resource allocation. This article mainly focuses on computing offloading decision-making, that is, whether to offload, what to offload, and where to offload for users. Liu et al. have developed a dynamic unloading strategy. Unloading is considered a two-stage stochastic optimization problem. From a standalone model, the cell phone uses Markov's method to determine whether to work internally or via a MEC server. To solve this problem, we provide single-bit research to solve the problem of power limit latency [5]. Lin et al. have been pursuing a goal of efficiency, providing a self-saving energy MEC system and a strategy for online accounting to get a good solution [6]. Zhu solved the problem of unloading one job of MEC; there are hundreds of cell phones and sensors needed to unload the load on industrial production lines, and a distribution strategy requires the unloading position [7]. Yanan et al. considers unloading tasks from another aspect, mainly for a series of tasks with sequential relationships, unloading through the optimization of the topology map and using load balancing heuristics to unload tasks to the MEC to maximize mobility and parallelism between a device and the cloud [8]. Other studies have also proposed the Hungarian algorithm to solve some nonsequential tasks, which generally require local equipment for preliminary processing. MEC completes subsequent high-computational tasks and also provides a new method in parallelism between mobile devices and the cloud. Chen et al. modeled the multiuser multi-MEC scenario as an energy optimization problem under the condition of delay constraints and solved the decision vector using the AFSA [9]. Alkhalaileh et al. proposed a fast hybrid multisite computing offload solution based on cloud computing, which could achieve optimal and near-optimal offload partitions according to the size of the mobile application to get a very suitable uninstall optimization solution [10]. Zhao et al. proposed a mobile device computing offload strategy based on Long Short-Term Memory (LSTM) network to predict computing tasks, combining with artificial intelligence technology. At present, various technologies tend to integrate with each other to achieve better results and use neural networks or machine learning to assist in optimizing the edge computing offloading model [11]. Huang summarized the research on computing offloading strategies in recent years, mainly according to the offloading types of computing offloading and optimization objectives and proposed solutions, scenarios, and evaluation methods for classification and summary. The possible application directions of MEC in the future will mainly focus on dynamic content optimization, Internet of Things, mobile big data analysis, and intelligent transportation [12].

RETRACTED

Based on the current research, this article proposes a method based on the PSO algorithm in the edge computing environment. PSO calculates and simulates bird flock foraging activities, the Frank Heppner biological group model, and the three rules in bird activities. After studying the activities of these natural creatures, abstract problems are quantified and similar models are established. The Gini coefficient is calculated by using grouped data, and the basis for grouping is also innovative. The quantile grouping method is adopted, which can effectively solve the difference between the concentration index and the Gini coefficient, and the Gini coefficients of each year can be added to finally get the Gini coefficient of the stock income.

## 3. Research on Optimal Scheduling Algorithm

The swarm intelligence algorithm is used to solve the optimal target of the problem by simulating the foraging activities of a biological group. This kind of algorithm has attracted more and more attention because of its simple principle and the advantages of quickly solving the target. With the continuous improvement and development of optimization algorithms, many swarm intelligence algorithms have been widely used, among these the most widely used algorithms mainly include ant colony, particle swarm, and artificial fish swarm methods and genetic algorithm (Figure 2) [13].

Because the principle of particle swarm optimization is simple, the calculation speed is fast, and considering that the research problem in this article is a discrete problem, this article chooses the particle swarm optimization to study the optimization problem.

The PSO algorithm simulates bird flock foraging activities, the Frank Heppner biological population model, and the three rules in bird activities. After studying the activities of these natural creatures, abstract problems are quantified and similar models are established. Later, other experts have improved and developed the models on this basis such that the performance of the algorithm has been continuously improved, the application fields have become more and more extensive, and many engineering problems have been solved [14].

RETRACTED

When solving problems, the PSO algorithm is simple and easy to understand. There is no complex function formula derivation or formula calculation. The model can be realized by setting a few parameters. On this basis, only a fitness function is needed to use the algorithm to optimize the target. The algorithm is similar to the genetic algorithm in that it sets the initial conditions, iterates many times to find the target, and uses the fitness to evaluate whether the solution target is achieved. Different from the genetic algorithm, the PSO algorithm does not require to go through complex crossover mutation like the genetic algorithm and directly searches for the optimal target until the optimal target is found.

### 3.1. Basic Particle Swarm Optimization

The principle of the PSO algorithm is the solution process in which each particle representing the solution of the problem continues to iteratively seek the optimal solution within a search range. The fitness generally represents the objective function problem we want to solve, and the optimal result of the problem is found through the objective function problem. What needs to be considered in this process is the speed and direction of the particles. The solution process of the algorithm is the process of continuous iteration of particles to find the optimal value. In a D-dimensional target search space, the initial number of particles is set to *m* [15]. The velocity and position update formulas are as follows:

(1) $$\begin{array}{c} v_{id+1}=wv_{id}+c_{1}\times \text{rand}\left(\right)\times \left(p_{id}-x_{id}\right)+c_{2}\times \text{rand}\left(\right)\times \left(p_{gd}-x_{id}\right), \end{array}$$

(2) $$\begin{array}{c} x_{id+1}=x_{id}+v_{id}+1, \end{array}$$

(3) $$\begin{array}{c} v_{id}=\left\{\begin{array}{cc} v_{\max}, & v_{id}>v_{\text{max}},\\ -v_{\max}, & v_{id}<v_{\text{max}},\\ v_{id}, & \left|v_{id}\right|<v_{\text{max}}. \end{array}\right. \end{array}$$

Among these, the position of the i-th particle in the d-th dimension is expressed as *x*_*id*_, the speed setting is expressed as *v*_*id*_, the current optimal position of the particle is expressed as *p*_*id*_(*p* Best), and the global optimal position of the particle is expressed as *p*_*gd*_(*g* Best). The inertia weight factor is represented as *w*, where *w* generally takes 1, rand ( ) represents a random number between [0, 1], and *c*_1__and_*c*_2_ represent the learning factors. The velocity range set by the particles in the process of continuous iteration is (*v*_min_, *v*_max_).

RETRACTED

Since the parameters of particle swarm optimization have different effects on the convergence of the algorithm, the correct setting of the algorithm parameters will help to improve the search and convergence performance of the algorithm (Figure 3).

#### 3.1.1. Particle Range

Since different problems have different fitness functions, the particle range is also different, but there will be a constraint range.

#### 3.1.2. Particle Scale

The size of the particle reflects the size of the search space of the algorithm. When the particle size is larger, the search space of the algorithm is larger, and vice versa, so the particle size should be selected in an appropriate range [16].

#### 3.1.3. Maximum Particle Speed

When using the algorithm to solve the target problem, the particle swarm algorithm achieves the solution of the optimal target by continuously updating the position of each particle. The search speed of the particle affects the search range of the particle. If the particle speed is set too large, it may cause the particle to fly. It is invalid if it goes out of the search space, so the maximum speed of the particles should be controlled within a reasonable range.

#### 3.1.4. Learning Factor

When the algorithm solves the problem, the learning ability of the particles in the iterative process is determined by the learning factors *c*_1_ and *c*_2_. The particles learn a kind of experience information through the speed, direction, and comparison with the optimal position, and then change their positions through this experience information such that they get closer and closer to the optimal target. *c*_1_ represents the learning ability of self-experience information and *c*_2_ represents the learning ability of social experience information. If *c*_1_ is larger, it will cause the particle to wander locally, and if *c*_2_ is larger, it will cause the particle to converge prematurely. Therefore, the size setting of the learning factors affects the quality of the solution target. In order to achieve an effective balance between the global search and local search, *c*_1_ and*c*_2_ should be set reasonably. Usually, the two take the same value of *c*_1_ and *c*_2_.

### 3.2. Improved Particle Swarm Algorithm

#### 3.2.1. Inertia Weight Factor Improvement Method

The inertia weight also has an important influence on the result of solving the target. Therefore, in order to improve the effect of solving the target, there have been many previous studies on the weight factor. The weight factor is set to various numbers that are constantly changing to realize the search of the optimization process. At present, the inertia weight factor is usually set as a function that changes with the number of iterations. Generally, there are these following situations:

(4) $$\begin{array}{c} w_{1}\left(k\right)=\frac{w_{\text{start}}-\left(w_{\text{start}}-w_{\text{end}}\right)\left(T_{\text{max}}-k\right)}{T_{\text{max}}}, \end{array}$$

(5) $$\begin{array}{c} w_{2}\left(k\right)=w_{\text{start}}-\left(w_{\text{start}}-w_{\text{end}}\right){\left(\frac{k}{T_{\max}}\right)}^{2}, \end{array}$$

(6) $$\begin{array}{c} w_{3}\left(k\right)=w_{\text{start}}-\left(w_{\text{start}}-w_{\text{end}}\right)\left[\frac{2k}{T_{\max}}-{\left(\frac{k}{T_{\max}}\right)}^{2}\right]. \end{array}$$

From Figure 4, it can be seen that in formula 3, the rate of change of *w* is from large to small, and the value is large at the beginning, which ensures the ability of the algorithm to search globally. After that, the rate of change gradually increases and the local optimization of the algorithm becomes better. This method can well balance the global search and local search capabilities and achieve better optimization results than by the fixed value of *w* [17].

RETRACTED

#### 3.2.2. Learning Factor Improvement Method

The learning ability in the particle optimization process is determined by the learning factors *c*_1_ and*c*_2_. If the value of *c*_1_ is large, it is easy to make the particle fall into the local area, and if the value of *c*_2_ is large, the particle will fall into the local optimum very early. In order to balance the global and local search capabilities, the compression factor method model constructed in it has better performance improvement in the convergence of the algorithm. The principle of this method is to improve the algorithm by adjusting the learning factors. The principle formula is specifically expressed as follows:

(7) $$\begin{array}{c} v_{id}^{k+1}=\phi \left(v_{id}^{k}+c_{1}r_{1}\left(p_{id}^{k}-x_{id}^{k}\right)\right)+c_{2}r_{2}\left(p_{gd}^{k}-x_{id}^{k}\right). \end{array}$$

(8) $$\begin{array}{c} \phi =\frac{2}{\left|2-C-\sqrt{C^{2}-4C}\right|}. \end{array}$$

Among these, *ϕ* represents the shrinkage factor, *C*=*c*_1_+*c*_2_, and C > 4, generally *ϕ*=4.1, and in this case, *c*_1_=*c*_2_=2.05.

#### 3.2.3. Algorithm Performance Test

In order to test the performance of the PSO algorithm before and after the algorithm improvement, this section selects the Griewank function:

(9) $$\begin{array}{c} f\left(x\right)=\frac{1}{4000}\sum_{i=1}^{n}x_{i}^{2}-\text{cos}\frac{x_{i}}{\sqrt{i}}+1, \end{array}$$

(10) $$\begin{array}{c} f\left(x\right)=\frac{1}{4000}\sum_{i=1}^{n}x_{i}^{2}-\cos\frac{x_{i}}{\sqrt{i}}+1. \end{array}$$

As a test function, the minimum value of the function is solved, and then the simulation test is carried out. The parameter settings are as follows: the number of iterations is set to 2000, the dimension is 10, the particle size is set to 30, the weight factor of the PSO algorithm before the improvement is set to a fixed value *w* = 0.7298, the learning factor is set to *c*_1_=*c*_2_=1.4962, and the weight factor of the improved PSO algorithm is set to wI (k); the value of the learning factor derived using the method described above is set to *c*_1_=*c*_2_=2.05.

RETRACTED

Based on the algorithm before and after the improvement, the convergence results of the test function are obtained respectively, and the convergence results are compared. From the final convergence results in Figure 5, it can be concluded that the convergence results before and after the improvement of the algorithm are 0.0393 and 0.0083, respectively. It can be seen that the performance of the unimproved PSO algorithm is not as good as that of the improved algorithm in terms of the convergence speed and the convergence results. It has been verified by simulation experiments that the improved PSO algorithm has better results in terms of convergence speed and convergence results [18].

Therefore, the improved PSO algorithm is selected to solve the subsequent problems. The steps of the PSO optimization algorithm to solve the optimal target are shown in Figure 6.

1. Initialize particles
2. Initialize the initial velocities and positions of N particles.
3. Calculation of fitness value
4. The function or equivalent function of the problem is selected as the fitness function in the solving process, and then the fitness value is solved according to this function.
5. Find the individual optimal fitness value
6. Compare the pBest (historical optimal position) of each particle with the current position of the fitness rate and determine whether to change the particle optimal position according to the particle fitness value. If the exercise rate is good, transfer the current material to a visible free particle.
7. Find the best value for the strong team
8. The process is similar to the previous steps. The fitness rate of gBest (the best in the world) for all is compared and the particle fitness rate is determined by whether the optimal particle position is adjusted [19].
9. Particle position and velocity update
10. After the abovementioned comparison of the fitness values, the position and velocity of the particle are updated according to the expression of the correlation function.
11. Judging whether to end
12. According to the set number of iterations, if the condition is not met, continue the iteration from the second step, otherwise, end the iteration, and gBest is the global optimal solution.

RETRACTED

### 3.3. Calculation of Gini Coefficient

The Gini coefficient is independent of the general entropy index, so this section briefly introduces several main calculation formulas of the Gini coefficient. This article mainly discusses how to measure the income gap of stock income, that is, to add the Gini coefficients of each year. Due to the extensive and in-depth research on the Gini coefficient, this article selects the Gini coefficient as an indicator to measure the stock income gap. At present, there are many methods for calculating the Gini coefficient, and the emphasis of each calculation method is different.

On the basis of the absolute average difference, the calculation method of the Gini coefficient is given as

(11) $$\begin{array}{c} G=\frac{\Delta_{n-1}}{2\mu }=\frac{1}{2n\left(n-1\right)\mu }\sum_{i=1}^{n}\sum_{i=1}^{n}\left|x_{i}-x_{j}\right|. \end{array}$$

According to the calculation formula of Gini coefficient and the consistency of covariance, the covariance formula of Gini coefficient is given as

(12) $$\begin{array}{c} G=\frac{2\text{ cov}\left(x_{i},i\right)}{n\mu }. \end{array}$$

Equations (11) and (12) are calculation formulas based on discrete income data. As shown in Figure 7, we assume that the income data obeys a continuous distribution function, and we introduce the analysis method of the Lorenz curve. Assuming that *x* is an income variable, its cumulative distribution function is F(x), and we take F(x) as the abscissa and the income L(x) owned by everyone whose income is not greater than *x* as the ordinate. The points connect to form a Lorenz curve, where *F*(*x*) = ∫_*x*_0__^*x*^*f*(*t*)*dt*, *L*(*x*) = 1/*μ*∫_*x*_0__^*x*^*tf*(*t*)*dt*.

From this, we can obtain the Gini coefficient calculation formulas (13–15) under the continuous distribution. After identity transformation, the following calculation formulas can be obtained:

(13) $$\begin{array}{c} G=1-2\int_{a}^{b}L\left(x\right)dF\left(x\right), \end{array}$$

(14) $$\begin{array}{c} G=\frac{1}{\mu }\left[\int_{a}^{b}F\left(x\right)\left(1-F\left(x\right)\right)\right], \end{array}$$

(15) $$\begin{array}{c} G=1-\frac{1}{\mu }\left[\int_{a}^{b}{\left(1-F\left(x\right)\right)}^{2}\right]. \end{array}$$

Since the “China Statistical Yearbook” uses grouped data to count income data, it is of great practical significance to calculate the Gini coefficient under the condition of grouped data. The calculation of the Gini coefficient of grouped data is based on the calculation formula of continuous data. The income data sample is divided into several groups, the income share owned by each group is calculated, and then the Lorenz curve is constructed, so that the Gini coefficient can be obtained [20].

RETRACTED

## 4. Simulation Experiments

The research time span of this article has been long; this article uses the income survey data in the “China Statistical Yearbook 2001–2019”; and the income survey data of the past years are presented in the form of grouped data.

Under the condition of grouped data, the estimation methods of moment estimation and maximal estimation cannot estimate parameters well. In addition, the distribution functions used to describe income data are nonlinear, and the quantile estimation methods cannot be well estimated. To estimate the parameters of income distribution, it is necessary to change the way of thinking in choosing the income distribution function and estimation method. The classical mathematical analysis theory holds that the function f(x) has an (*n* + 1) order derivative in a certain neighborhood, then the function can be expressed as *f*(*x*) = ∑_*n*=0_^*∞*^*f*^(*n*)^(*a*)/*n*!(*x* − *a*)^*n*^*𝔐*, which is also called the Taylor series [21]. For distribution functions such as normal distribution, logistic distribution, gamma distribution, and Dagum distribution, there are (*n* + 1) order derivatives, so the distribution function can use Taylor series expansion and convert the distribution function into a polynomial. Under the condition of known quantiles, a polynomial curve can be obtained by interpolation, which is consistent with the polynomial of the distribution function expanded by the Taylor series, so it is very easy to solve. This avoids the controversy over the choice of distribution function types and can achieve a good estimation effect. The income data obtained in this article are urban and rural grouped data, therefore the interpolation method is used to estimate the urban and rural income distribution functions, respectively. According to the obtained income distribution function over the years, we calculated the Gini coefficient of urban and rural areas separately. Then, using the method of random simulation the income data are generated according to the population size of towns and villages and the Gini coefficient of the whole country is calculated; finally, the Gini coefficient of assets is calculated according to the Gini coefficient of the whole country from past years to evaluate the inequality of asset distribution [22].

### 4.1. Interpolation Calculation: Urban and Rural Income Distribution Function

Judging from the current research progress, the algorithm theory of interpolation is relatively mature. According to the form of the interpolation function, it is mainly divided into algebraic polynomial interpolation, triangular polynomial interpolation, and rational fractional interpolation. Algebraic polynomial interpolation is the most commonly used interpolation method. It is also the most abundantly used, which mainly includes equidistant node interpolation, nonequidistant node interpolation, piecewise interpolation, and reverse interpolation, which maximizes the number of iterations. The accuracy of the above methods is very close. The income accumulation can be obtained by interpolation calculation, and the distribution function *F*_*c*_(*x*) = ∑_*i*=1_^*m*^*c*_1*i*_*x*^*i*^ can be calculated. Using the same calculation method, the inverse function *F*_*c*_^−1^(*p*) = ∑_*i*=1_^*n*^*y*_1*i*_*p*^*i*^ of the income distribution function can be calculated. In this way, the income distribution function of urban residents can be obtained. Compared with the distribution function estimated directly by the moment estimation method or the point estimation method, the income distribution function obtained by the interpolation method has a high precision and overcomes the obstacles brought by grouped data to the moment estimation method and the point estimation method. Estimate the cumulative income distribution function of rural residents. The statistical method used for the rural residents' income data is different from that of the urban residents' income data. The population proportion in a fixed interval is given, and the interpolation method is also used to estimate the income distribution function of the rural residents. *F*_*N*_(*x*) = ∑_*i*=1_^*m*^*c*_2*i*_*x*^*i*^and the inverse function *F*_*N*_^−1^(*p*) = ∑_*i*=1_^*n*^*y*_2*i*_*p*^*i*^ of the income distribution function, are the polynomial form of the number of urban residents in 2018, as shown in Equation (4)–(1) and Equation (4)–(2), a more intuitive expression is shown in Figures 8 and 9. As can be seen from Figures 8 and 9, the income distribution function in the polynomial form can estimate the income distribution function well and the estimation accuracy can be guaranteed, and its effect is far better than the type of the selected income distribution function [23]. With regard to the effect of grouped data estimation, this estimation method is difficult to match with the other estimation methods.

(16) $$\begin{array}{c} F_{C}^{2018}\left(x\right)=-0.2789\times 10^{-28}x^{6}-0.9061\times 10^{-24}x^{5}+0.1124\times 10^{-17}x^{4}-0.1124\times 10^{-12}x^{3}+0.3804\times 10^{-8}x^{2}-0.1773\times 10^{-4}x+0.1152\times 10^{-2}, \end{array}$$

(17) $$\begin{array}{c} F_{N}^{2018}\left(x\right)=0.1179\times 10^{-24}x^{6}-0.1022\times 10^{-19}x^{5}+0.3462\times 10^{-15}x^{4}-0.5649\times 10^{-11}x^{3}+0.4114\times 10^{-7}x^{2}-0.2586\times 10^{-4}x+0.4112\times 10^{-4} \end{array}$$

RETRACTED

### 4.2. Measurement of Stock Income Gap and Analysis of Influencing Factors

Due to the lack of consumption data in the income data released by the Bureau of Statistics, the current stock income gap in China cannot be accurately measured. In order to grasp the current gap between traffic and income in China at a macro level, we directly calculated the Gini coefficient of stock income on the basis of the Gini coefficient of traffic income. Although this underestimates the current stock income gap, the results are still useful for studying the current stock income gap. The Lorenz curve and Gini coefficient can be further obtained according to the polynomial, and the relationship between the Lorenz curve and income distribution function can be obtained from the definition of the Lorenz curve, as shown in formula (18), and then the distribution integration method is used for identity transformation.

(18) $$\begin{array}{c} L\left(x\right)=\frac{1}{\mu }\int_{0}^{x}tf\left(t\right)dt=\frac{1}{\mu }\int_{0}^{x}t\;dF\left(t\right)=\frac{1}{\mu }\left(tF\left(t\right)|0_{x}-\int_{0}^{x}F\left(t\right)dt\right)=\frac{1}{\mu }\left(xF\left(x\right)-\int_{0}^{x}F\left(t\right)dt\right). \end{array}$$

As shown in Figure 10, the Gini coefficients of rural, urban, and national stock incomes all show an upward trend. By 2018, the Gini coefficients of the national stock incomes had risen to 0.4378. In Figure 10, both the national Gini coefficient and the Gini coefficient of stock income show an overall upward trend. Although the Gini coefficient of traffic income had declined in 2017 and 2018, there has been no obvious decline in the stock income. As discussed in Section 3.3, there is inertia in the stock income gap. Therefore, the current income gap is relatively large, and we hope to narrow the income gap in the future, but the policy effect of reducing the income gap in the future will be discounted and will not have an immediate effect. Even though the flow-income gap has dropped significantly, the range of changes in the stock value is relatively small [24].

Calculated from the income distribution function, the Gini coefficient of urban residents' income in 2018 was 0.3310 and the Gini coefficient of the residual income after consumption adjustment was 0.4048, with an increase of 22.27%—a large increase. Use the same method to calculate the Gini coefficient and the Gini coefficient of residual income for other years, as shown in Figure 11 and Figure 12. It can be seen from Figures 11 and 12 that the difference between the Gini coefficient of residual income and the Gini coefficient of income is large. The Gini coefficient of residual income is significantly larger than that of income, but the increase has a downward trend year by year. It is intuitively reflected from the graph that the consumption expenditure has widened the income gap. In 2002, consumption increased the Gini coefficient by 80.38%, while in 2018, the Gini coefficient of residual income increased by 22.27% as compared with that of income. Since income from investment is included in the data released by the Bureau of Statistics, it is impossible to disentangle investment data to analyze the effect of investment on the widening income gap [25].

RETRACTED

In the above calculation, due to the lack of consumption data and investment data, the influence of consumption and investment on the cumulative income distribution function was not evaluated. On the basis of the previous section, the impact of consumption on the stock income gap is assessed based on the urban income data from 2002 to 2018. According to the definition of the stock income gap, the consumption is first deducted from the income and then the remaining income is added to the investment income to obtain the final annual income flow. Since only the urban income data from 2002 to 2018 can be obtained at present, the income data of 17 years is used as a sample to observe the impact of income consumption on the stock income gap. According to the calculation method of the stock income gap, the calculation results of the stock income gap after consumption adjustment are shown in Figure 13, Figure 14, Figure 15, and Figure 16. From the calculation results, the Gini coefficients of the four types of income all show an upward trend, and after 2015, they decreased slightly; from the perspective of the residual income gap and the stock residual income gap, the inertia is more prominent, and for the residual income from 2015 to 2018, the Gini coefficient had dropped significantly, but the stock residual income had not dropped significantly [26].

From Figure 17, Figure 18, Figure 19, and Figure 20, we can conclude that the adjustment direction of the Gini coefficient of stock income and the Gini coefficient of income flow is the same, but when stock income accumulates to a certain extent. The Gini coefficient of traffic income in 2017 and 2018 had dropped significantly, but the change in the Gini coefficient of stock income (Delta CG) was still greater than 0. Obviously, the speed of adjustment is lagging behind the Gini coefficient of traffic income, which is the so-called lag. The facilitation effect is greater than the dilution effect, and the facilitation effect continues to push up the stock income gap, which indicates more income flows to the high-income group and rising traffic income gap, with the upward trend becoming more and more obvious. With the passage of time, the stock income gap becomes more difficult to be changed by the income flow gap. It becomes more and more difficult to narrow the real stock income gap in the future. Therefore, we cannot pin the hope of narrowing the income gap on the future. The stock income gap of China cannot be narrowed overnight, and it requires sustained and continuous efforts to be achieved.

RETRACTED

## 5. Conclusion

We analyzed and studied the solution method of multiobjective problems, the principle and characteristics of the standard PSO algorithm, and the principle and characteristics of the improved PSO algorithm on this basis. In order to study the income gap of stock income, the additivity of the Gini coefficient must be studied, which is inherently consistent with the decomposition of the Gini coefficient by income source. In order to overcome the obstacle caused by the pseudo-Gini coefficient, the quantile is used as the basis for grouping such that the obstacle can be effectively overcome and the Gini coefficients of different years be added. Research shows that the Gini coefficient of stock income is the weighted value of the Gini coefficient of income flow, and the weight is the proportion of the total income of each year to the total income of all years.

To sum up, there is a long way to go in the work of adjusting the income gap in the future. The diversification of residents' income composition is the main reason for the uncontrollable income gap. Before the reform and opening up, labor income was the main source of income for residents, and after the reform and opening up, the ownership reform and distribution system reform allowed other production factors to participate in the distribution. In China with a large population, labor resources are abundant. By contrast, production factors such as capital and technology have become scarce resources. In this way, the marginal return of labor is low, and residents who only rely on labor to obtain income must be at a disadvantaged position in the current income distribution, which is the main reason for the widening of the gap between traffic and income. Looking at the income data of the past years, the per capita income shows a trend of continuous growth, but the growth trend of various incomes is different. The proportions have increased. The current distribution policy is based on the distribution according to work, supplemented by distribution according to production factors. For low-income people, labor is the main way to obtain income, while for high-income people, labor is only one of the ways of sources of income. For China with a large population, labor resources are abundant. Relatively speaking, capital has become a scarce resource. From the perspective of supply and demand, the price of capital is greater than the price of labor.

RETRACTED

## Figures and Tables

**Figure 1:** Edge computing core technology.

**Figure 2:** Performance comparison of several swarm intelligence algorithms.

**Figure 3:** Particle position update process.

**Figure 4:** Changes of several weighting factors.

**Figure 5:** Test results before and after the improvement of the PSO algorithm.

**Figure 6:** Particle swarm algorithm flow.

**Figure 7:** Lorenz curve.

**Figure 8:** Empirical distribution and polynomial income distribution function of urban income data in 2018.

**Figure 9:** Empirical distribution and polynomial income distribution function of rural income data in 2018.

**Figure 10:** Gini coefficient of income flow and Gini coefficient of stock income (1985–2018).

**Figure 11:** Income Gini coefficient and residual income Gini coefficient of urban residents.

**Figure 12:** Adjustment width.

**Figure 13:** Gini coefficient.

**Figure 14:** Gini coefficient of stock income.

**Figure 15:** Gini coefficient of residual income.

**Figure 16:** Gini coefficient of stock residual income.

**Figure 17:** Gini change in stock income (Delta CG).

**Figure 18:** Gini change in traffic income (Delta FG).

**Figure 19:** Promotion effect.

**Figure 20:** Dilution effect.

## Data Availability

The labeled dataset used to support the findings of this study are available from the corresponding author upon request.
